# J Point and ST Elevation Resembling Brugada: A Marker of Mortality in Methanol Toxicity

**DOI:** 10.1155/2021/5541385

**Published:** 2021-07-19

**Authors:** Mohammad Hossein Nikoo, Alireza Estedal, Kiana Khatami, Maryam Pakfetrat, Alireza Arjangzadeh, Shahrokh Sadeghi Boogar, Sina Danesh, Seyed Taghi Heydari

**Affiliations:** ^1^Non-Communicable Disease Research Centre, Shiraz University of Medical Sciences, Shiraz, Iran; ^2^Health Policy Research Center, Institute of Health, Shiraz University of Medical Sciences, Shiraz, Iran; ^3^Department of Internal Medicine, Shiraz Nephro-Urology Research Center, Shiraz University of Medical Sciences, Shiraz, Iran; ^4^Cardiology Department, Shiraz University of Medical Sciences, Shiraz, Iran; ^5^Department of Internal Medicine, School of Medicine, Shiraz University of Medical Sciences, Shiraz, Iran

## Abstract

**Objective:**

*J* point and coved ST elevation in right precordial leads (not produced by coronary artery disease) are still a matter of challenge, especially when resembling Brugada patients. This clinical entity, among asymptomatic individuals with no family history of sudden cardiac death, would be reported in some severely ill patients before ventricular fibrillation. This study investigated the relationship between the electrocardiograms with demographic and laboratory data and also analyzed their association with mortality rate among patients with methanol poisoning.

**Methods:**

The sample consisted of 356 patients who were hospitalized with a diagnosis of methanol poisoning in Faghihi and Namazi Hospitals in Shiraz, Southern Iran, in March and April 2020. In this period, a major outbreak of methanol poisoning had occurred in this area. Furthermore, the study used the data on any recorded complications or mortality during hospital course.

**Results:**

The ECG (BrP) was observed in a total of 20 (5.6%) patients. Its presence was associated with increased mortality, Glasgow coma scale score <3, and blood sugar levels and was inversely associated with PH, O_2_ saturation, and calcium levels (*P* < 0.05).

**Conclusions:**

This study found that certain ECG patterns and laboratory data can be used as prognostic factors of morbidity and mortality in patients with methanol intoxication. Electrocardiography machines are widely available tools, which can be easily used for risk stratification based on the presence of Brugada approximating electrocardiograms among patients with methanol intoxication.

## 1. Introduction

Brugada syndrome (BrS) is an autosomal dominant genetic disorder with variable expressions characterized by abnormal findings on the standard 12-lead electrocardiogram (ECG). This syndrome is associated with an increased risk of ventricular tachyarrhythmias and sudden cardiac deaths [1]. Brugada phenocopies are recently introduced as clinical entities with electrocardiographic patterns identical to the true congenital Brugada syndrome in individuals who are asymptomatic and have no other clinical criteria, especially if the typical pattern is resolved after improvement of the patient's condition [2, 3]. These Brugada ECG patterns are present in various clinical conditions such as myocardial ischemia and diseases, mechanical chest compression, pulmonary embolism, electrolyte imbalances, and metabolic derangements and are provoked by the administration of special medications [2, 4–6].

Methanol (also known as methyl alcohol, wood alcohol, wood spirits, and carbinol) is a widely available chemical in industries, and it is also present in a number of household products, including varnish, windscreen washer fluid, and antifreezes. Methanol has a relatively low intrinsic toxicity; however, it is metabolized in human body and converted to highly toxic compounds such as formaldehyde, formic acid, and format [7]. These metabolites can cause blindness, coma, and life-threatening metabolic disturbances. Owing to the delayed effects of these toxic metabolites, patients do not often come to clinical attention in a timely manner, resulting in high rates of morbidity and mortality in the outbreaks of methanol poisoning.

Outbreaks of methanol poisoning often occur due to erroneous techniques as part of the illicit manufacture of alcoholic drinks [8, 9]. Because patients with methanol poisoning often need intensive medical care, outbreaks of methanol poisoning can rapidly overwhelm medical facilities. In March and April 2020 in Iran, a major methanol outbreak occurred in the wake of the COVID-19 pandemic, resulting in an extensive death toll of about 534 persons throughout the country based on Iran's Health Ministry Spokesman and Iranian Legal Medicine Organization (LMO) [10]. Among the provinces, Fars had the highest reported number of patients with methanol toxicity [11].

Recent literature has described an association between BrP and mortality. This study adds to these literatures by a detailed examination of 20 methanol-intoxicated patients with this ECG pattern and the association of this finding with mortality. Monterrubio-Villar et al. [12] in a case report presented a 54-year-old man with the extreme metabolic acidosis and a Brugada type 1 ECG pattern, which later led to the patient's brain death. Jaff et al. [13] reported a type one Brugada ECG pattern in a patient concurrently sedated with an infusion of propofol who later developed permanent neurologic damage and expired. This study shed more light on the Brugada phenocopy by describing a detailed examination of 20 patients who presented with Brugada ECG pattern and highlighted the significance of this finding as a mortality marker.

## 2. Methods

Data were collected from 356 patients who were diagnosed with methanol poisoning and were hospitalized in Faghihi and Namazi Hospitals in Shiraz, southern Iran, in March and April 2020. These two major tertiary-care hospitals are affiliated to Shiraz University of Medical Sciences. Some poisoning care referral centers were designated at these hospitals during the aforementioned methanol toxicity outbreak. The study extracted the demographic data such as age, gender, medical history, Glasgow coma scale score, development of any complications such as decreased visual acuity or renal problems, and mortality during the hospitalization course from admission sheets. Laboratory data such as arterial blood gas data (pH, partial pressure of carbon dioxide (torr), bicarbonate (meq/L)), oxygen saturation (%), creatinine level (mg/dL), blood urine nitrogen level (mg/dL), blood sugar (mg/dL), and electrolyte variables, including sodium (meq/L), potassium (meq/L), magnesium (mg/dL), and calcium (mg/dL), were gathered using the HIS (Health Information System) of the affiliated hospitals.

BrP was diagnosed by identifying *J* wave elevation and coved ST elevation in right precordial leads *n* on a standard 12-lead electrocardiogram in the absence of a true congenital Brugada syndrome. Two forms of the Brugada ECG pattern are described: type 1 pattern has *j* point elevation ≥2 mm, “coved-type” ST segment, and an inverted *T* wave in V1 and V2 (Figure 1). Type 2 pattern has a “saddle-back” ST segment with at least 1 mm elevation [2, 14]. CARDIAX PC-ECG was used to obtain the electrocardiographic data, collected by a cardiologist. These ECGs were analyzed and reported independently by two cardiologists.

## 3. Statistical Analysis

Statistical Package for the Social Sciences (SPSS Inc., Chicago, IL, USA), Version 21.0, was used to analyze the data. Frequency (%) was used to describe the categorical variables such as gender, alcohol dependency, comorbidity, and BrP. Moreover, mean ± standard deviation was used to describe scale variables such as age and laboratory findings. Independent-samples *t*-test was used to compare the mean of the laboratory findings (i.e., PH, Hco3, Pco2, BUN, Cr, etc.) between patients with and without BrP. Chi-squared test was used to compare the frequency of previous cardiac and noncardiac diseases, death, renal failure, and decreased visual acuity between patients with and without BrP. *P* < 0.05 was considered statistically significant.

## 4. Results

A total of 20 (5.6%) patients were admitted with the diagnosis of methanol toxicity and concurrent Brugada similar patterns, among whom four (20.0%) patients had comparable type 1 and 16 (80.0%) patients had saddle-back ST elevation (like type 2). Interestingly, none of these patients had a history of medical diseases. Comparing the patients with and without BrP revealed that mortality rate (Brugada: 45.0%, non-Brugada: 13.5%, *P* < 0.001), renal failure (Brugada: 65.0%, non-Brugada: 34.3%, *P*=0.008), Glasgow coma scale score < 3 (Brugada: 35.0%, non-Brugada: 11.5%, *P*=0.008), and blood sugar (Brugada: 227.25 ± 124.15, non-Brugada: 139.17 ± 92.23, *P* < 0.001) were significantly higher in the former group. In addition, PH (Brugada: 7.01 ± 0.26, non-Brugada: 7.15 ± 0.21, *P*=0.006), O_2_ saturation (Brugada: 81.94 ± 13.70, non-Brugada: 91.04 ± 9.90, *P* < 0.001), and calcium (Brugada: 10.05 ± 1.34, non-Brugada: 9.53 ± 0.725, *P*=0.018) were lower in Brugada phenocopy patients compared to methanol toxicity patients with no Brugada ECG pattern (Table 1). No significant difference was observed between the two groups in terms of age, gender, medical history, decreased visual acuity, bicarbonate, partial pressure of CO_2_, creatinine, sodium, potassium, and magnesium.

In patients with type 1 BrP, potassium (7.05 ± 1.20, *P*=0.001) and blood sugar (278.75 ± 46.70, *P*=0.001) were higher, and oxygen saturation (69.75 ± 9.95, *P* < 0.001), PH (6.76 ± 0.083, *P* < 0.002), and calcium levels (9.50 ± 0.36, *P*=0.023) were lower in comparison to the other Brugada pattern types. Furthermore, no significant difference was observed between the two groups in terms of age, bicarbonate, partial pressure of CO_2_, blood urine nitrogen, sodium, potassium, and magnesium (Table 2).

## 5. Discussion

Brugada syndrome has originally been described as a distinct clinical and electrocardiographic syndrome characterized by ST elevation with successive negative *T* wave in the right precordial leads, predisposing patients to the risk of sudden cardiac death (SCD) due to ventricular fibrillation (VF) [15]. However, Brugada syndrome in fact encompasses a number of Brugada ECG patterns, observed in various clinical conditions, leading to the proposal of “Brugada phenocopy” by Riera et al [6]. However, Brugada syndrome and Brugada ECG patterns have posed a number of controversies around the casual role of genetic variants and their underlying pathophysiology.

Methanol is relatively nontoxic and causes mainly central nervous system sedation. However, profound toxicity can ensue when methanol is metabolized in vivo (i.e., oxidized, primarily by alcohol dehydrogenase (ADH)). Alcohol dehydrogenase oxidizes methanol to formaldehyde, and aldehyde dehydrogenase subsequently oxidizes formaldehyde to formic acid. The methanol metabolite formic acid accumulates after large ingestions resulting in a profound anion gap metabolic acidosis [9]. Then, this metabolic acidosis and subsequent hyperkalemia can decrease Na^+^ current magnitude through inactivating the cardiac Na^+^ channel [16–18]. It is noteworthy that the patients with methanol toxicity in this study had acidosis and hyperkalemia; thus the pattern presented in the ECGs is a multifactorial Brugada pattern [19, 20].

According to the present findings, the higher levels of acidosis were significantly associated with the presentation of Brugada ECG patterns. These findings are in line with the previous studies, further supporting the idea that external PH affects sodium channel function, resulting in acidosis-induced arrhythmias, and triggers Brugada syndrome and sudden cardiac deaths [17, 18, 21, 22]. In addition, the first putative mutations leading to Brugada syndrome were found in SCN5A, which encodes the cardiac sodium channel NaV1.5 [23]. The fact that the function of this subunit is attenuated by acidosis also supports our hypothesis, indicating that low PH can play a major role in Brugada phenocopy as well as Brugada syndrome.

Another finding was the higher proportion of patients with decreased level of consciousness among BrP, in comparison to the other patients. This is in consistency with similar case report on methanol poisoning [12]. Monterrubio-Villar described a case of a 54-year-old man with extreme metabolic acidosis, hyperkalemia, and a Brugada type 1 ECG pattern. Upon correction of metabolic derangements, the Brugada ECG pattern normalized. However, the patient developed signs of cerebral herniation followed by brain death and died on the first day of ICU admission. A review of the literature indicated that Brugada syndrome can be provoked in conditions with decreased brain function such as sleep [24], brain injury [25], prolonged intubation in Intensive Care Units (ICU), sedative drugs overdoses [26–28], and propofol anesthesia [6]. These findings cast doubt on the association between the decreased levels of consciousness and associated lower brain function with the presence of Brugada ECG patterns.

Moreover, it was observed that BrP patients had lower levels of serum calcium, which was in line with previous studies. This may be due to the fact that the mutated sodium channel impairs the function of sodium-calcium exchanger, thus leading to such an alteration [26].

Another noticeable finding was that, between the two types of Brugada ECG patterns, type 1 pattern was associated with more dramatic laboratory alterations. More severe acidosis, higher potassium and blood sugar levels, and lower calcium levels were more commonly observed in Type 1 Brugada ECG patterns. This finding can be the subject of further research, exploring the association between laboratory data alterations and the severity of ECG changes.

## 6. Limitations

To our knowledge, this is the first study to focus on BrP in methanol toxicity with a comprehensive clinical data and a large sample size. This study was not able to delineate the underlying mechanisms of the findings given the scarcity of literature in this area. Moreover, the nonexecution of a provocative test therefore represents a diagnostic limit. This study is a retrograde study concerning ECG change in methanol poisoning patients conducted in the first months of the COVID-19 pandemic. Therefore it was not feasible to perform provocative test as it was not routinely done for methanol poisoning patients and also due to the fact that almost all of the healthcare providers were dealing with COVID-19 patients and outpatient clinics were closed. Finally, we highly recommend performing the sodium channel blocker provocative test for the future studies addressing presentation of Brugada pattern in methanol poisoning patients.

## 7. Conclusion

This study indicated that Brugada ECG patterns can be used for early identification and risk stratification of patients with methanol toxicity. Given that, ECG can be used as a valuable tool for this purpose due to its wide availability, feasibility, and low cost. In addition, correction of acidosis, hypocalcemia, and hyperkalemia can be an additional measure to correct such a pattern and possibly reduce the associated risk; however, there is a need for further research. The correction of acidosis, hypocalcemia, and hyperkalemia can be a technique to reduce the pattern; however, there is a need for further research.

## Figures and Tables

**Figure 1:** Patient with type 1 Brugada pattern, before and after presentation.

**Table 1:** Association between Brugada phenocopies and demographic variables, past medical history, mortality, complication in hospital, and laboratory data.

		Brugada pattern		*P* value
		No	Yes	
Sex	Male	300 (84.3)	17 (85.0)	0.436
	Female	32 (9.0)	3 (15.0)	
Previous cardiac disease	No	307 (86.2)	19 (95.0)	0.234
	Yes	23 (6.5)	0 (0.0)	
Previous noncardiac disease	No	310 (87.1)	19 (95.0)	0.269
	Yes	20 (5.6)	0 (0.0)	
Statutes	Live	279 (78.4)	11 (55.0)	<0.001
	Death	48 (13.5)	9 (45.0)	
Renal failure	No	202 (56.7)	6 (30.0)	0.008
	Yes	122 (34.3)	13 (65.0)	
Decreased visual acuity	No	87 (24.4)	3 (15.0)	0.274
	Yes	233 (65.4)	16 (80.0)	
GCSS	3	41 (11.5)	7 (35.0)	0.008
	4–14	42 (11.8)	4 (20.0)	
	15	242 (68.0)	9 (45.0)	
Age		32.51 ± 10.59	35.45 ± 9.59	0.226
PH		7.15 ± 0.21	7.01 ± 0.26	0.006
Bicarbonate (meq/l)		11.32 ± 8.12	8.86 ± 6.36	0.196
Partial pressure of carbon dioxide (torr)		27.89 ± 13.90	25.13 ± 11.42	0.398
Oxygen saturation (%)		91.04 ± 9.90	81.94 ± 13.70	<0.001
Creatinine (mg/dl)		1.420 ± 0.63	1.61 ± 0.60	0.208
Blood urea nitrogen (mg/dl)		14.00 ± 10.39	17.37 ± 17.05	0.189
Calcium (mg/dl)		9.53 ± 0.725	10.05 ± 1.34	0.018
Magnesium (mg/dl)		2.39 ± 1.60	2.67 ± 0.63	0.582
Sodium (meq/l)		142.1 ± 84.21	141.8 ± 44.09	0.734
Potassium (meq/l)		4.82 ± 1.13	4.91 ± 1.90	0.755
Blood sugar (mg/dl)		139.17 ± 92.23	227.25 ± 124.15	<0.001

**Table 2:** Comparison of age and laboratory data between various types of Brugada phenocopies.

	Brugada type			*P* value
	No	1	2	
Age	32.51 ± 10.59	31.75 ± 10.28	36.38 ± 9.54	0.354
PH	7.15 ± 0.211	6.76 ± 0.083	7.08 ± 0.26	0.001
Bicarbonate (meq/l)	11.31 ± 8.12	5.35 ± 2.49	9.79 ± 6.80	0.268
Partial pressure of carbon dioxide (torr)	27.89 ± 13.90	34.62 ± 12.08	22.6 ± 10.19	0.210
Oxygen saturation (%)	91.04 ± 9.90	69.75 ± 9.95	85.69 ± 12.69	<0.001
Creatinine (mg/dl)	1.41 ± 0.63	2.450 ± 0.26	1.39 ± 0.45	0.005
Blood urea nitrogen (mg/dl)	13.61 ± 7.63	14.25 ± 5.32	13.2 ± 4.86	0.964
Calcium (mg/dl)	9.53 ± 0.72	9.50 ± 0.36	10.21 ± 1.49	0.023
Magnesium (mg/dl)	2.40 ± 1.60	3.45 ± 0.21	2.48 ± 0.54	0.630
Sodium (meq/l)	142.1 ± 84.21	141.00 ± 6.98	142.07 ± 3.28	0.853
Potassium (meq/l)	4.82 ± 1.13	7.05 ± 1.20	4.30 ± 1.61	0.001
Blood sugar (mg/dl)	139.17 ± 92.23	278.75 ± 46.70	210.08 ± 138.33	0.001

## Data Availability

The Excel data used to support the findings of this study are available from the corresponding author upon request.
